# Magnetic Resonance Imaging under Image Enhancement Algorithm to Analyze the Clinical Value of Placement of Drainage Tube on Incision Healing after Hepatobiliary Surgery

**DOI:** 10.1155/2022/9269695

**Published:** 2022-05-31

**Authors:** Shihai Yang, Qihua Wu, Qi Wang, Fajin Lv

**Affiliations:** ^1^Department of Radiology, The First Affiliated Hospital of Chongqing Medical University, Chongqing 400016, China; ^2^Department of Radiology, Chongqing Nanchuan District People's Hospital, Chongqing 408400, China

## Abstract

This study was aimed at exploring the application value of magnetic resonance imaging (MRI) based on image enhancement algorithm in analyzing the placement of drainage tubes in the healing of incisions after hepatobiliary surgery. A total of 70 patients with liver cancer undergoing laparoscopic hepatobiliary surgery were selected, including 34 males and 36 females. According to the detection method of postoperative recovery, they were divided into a group A (conventional MRI detection) and a group B (MRI detection based on Retinex algorithm). Patients were divided into two groups according to whether subcutaneous drainage tubes were placed: group C (no subcutaneous drainage tubes were placed) and group D (subcutaneous drainage tubes were placed), with 35 patients in each group. The results showed that there was no significant difference between group A and group B in tumor residual or recurrence. The detection rate of tumor capsule in group B was significantly higher than that in group A (*P* < 0.05). The sensitivity, specificity, and accuracy of group A for the detection of recurrent lesions were 63.40%, 86.90%, and 78.60%, respectively; those in group B were 82.70%, 98.50%, and 93.20%, respectively. Therefore, the difference between the two groups was statistically significant (*P* < 0.05). The incidence of poor wound healing and infection in group C were significantly lower than those in group D (*P* < 0.05). Therefore, the effect of MRI detection based on image enhancement algorithm was more conducive to the evaluation of postoperative recovery due to the traditional MRI detection. In addition, the drainage tube was helpful to the postoperative wound healing and showed high clinical value.

## 1. Introduction

With the continuous improvement of China's basic living standards and the continuous improvement of living standards, coupled with the current fast pace of life and increased life pressure, the incidence of hepatobiliary surgery diseases (such as liver tumors and biliary stones) is constantly increasing [1]. Laparoscopic surgery is widely used in the treatment of hepatobiliary diseases because of its good therapeutic effect, and the evaluation of postoperative curative effect is related to the patient's prognosis and quality of life [2]. With the advancement of science and technology, various medical imaging technologies are constantly improving, and various new technologies and methods are gradually being applied to clinical diagnosis and treatment. Functional magnetic resonance imaging (fMRI) is a common product of molecular biology and medical physics and other related disciplines. It can dynamically detect the cells and molecules in the physiological and pathological processes of the organs and tissues in the patient's body in real time, realizing the diagnosis and monitoring treatment effect at the ultraearly highly specific pathological level [3]. The applications of fMRI in the liver mainly include magnetic resonance imaging (MRI), diffusion-weighted imaging (DWI), perfusion-weighted imaging (PWI), and magnetic resonance spectroscopy (MRS) [4]. MRI can keenly observe the changes in blood flow, energy, and metabolism of cells and has a very high ability to evaluate the curative effect and prognosis after surgery [5].

In computer-assisted diagnosis and treatment, medical image processing plays an auxiliary role that cannot be ignored [6]. Among them, medical image enhancement is an important part of image inspection [7]. Image enhancement technologies are mainly divided into two types according to the scope of the processing objects: enhancement methods based on frequency domain and enhancement methods based on spatial domain [8]. The object of the enhancement methods based on spatial domain is the gray value of the image, and the core is the selection strategy of the mapping transformation function [9], while the enhancement method based on spatial domain is to indirectly realize image enhancement by adjusting the transformation coefficients in the image transformation domain [10]. At present, the more common and typical image enhancement methods include histogram equalization and its improved algorithm, Retinex and its improved algorithm, wavelet transform method, morphology-based enhancement method, and fuzzy set-based image enhancement technology [11]. Among them, Retinex algorithm, histogram equalization, and image enhancement algorithm based on wavelet transform are widely used in medical images [12].

In addition, how to manage postoperative incisions in clinical treatment is critical to the prognosis of surgery. Once the incision infection occurs, it will take a longer time to treat, increase the patient's pain and economic burden, extend the hospital stay, reduce the turnover rate of hospital beds, and increase the workload of the doctor [13]. Therefore, subcutaneous negative pressure drainage tubes appear in the application of deep infection and plastic surgery. The working principle of drainage tubes is mainly relsiphon or negative pressure suction, and they are preset in the surgical area or body cavity of the human body; through the skin incision, the exudate and tissue fluid accumulated in the body tissue or body cavity are drained to the body to prevent fluid accumulation and cause postoperative wound infection, promoting wound healing and disease recovery [14]. This method is simple, easy, and low cost and can be used for all abdominal operations. Therefore, it has been clinically recognized and affirmed for use after many diseases. However, the discussions and disputes on drainage tubes are still unabated in domestic and foreign academic circles, and it needs to use a large number of clinical trials and experience to prove its effectiveness [15].

Therefore, liver cancer patients undergoing laparoscopic hepatobiliary surgery were selected as the research objects in this study. MRI based on Retinex algorithm was used to evaluate the treatment effect, which was compared with traditional MRI, to explore its application value in postoperative evaluation and the influence of drainage tubes on postoperative wound healing.

## 2. Research Methods

### 2.1. Research Objects

Seventy patients with liver cancer who received laparoscopic hepatobiliary surgery in hospital from June 2018 to June 2020 were selected and analyzed. There were 34 males and 36 females, with an average age of 54 ± 7.3 years. According to the postoperative evaluation method, they were divided into a group A (conventional MRI detection) and a group B (MRI detection based on Retinex algorithm). According to whether subcutaneous drainage tubes were placed, the two groups of patients were randomly divided into a group C (no subcutaneous drainage tubes were placed) and a group D (subcutaneous drainage tubes were placed), with 35 cases in each group. The patients included in the study had signed the informed consent forms, and the trial process had been approved by the ethics committee of hospital.

The inclusion criteria are as follows: the patients had complete case information; the patient was confirmed to be liver cancer by postoperative pathology; the diagnosis results conformed to the “five major six subtypes” classification and “primary liver cancer diagnosis and treatment standards” of the China Liver Cancer Pathology Research Collaborative Group. The exclusion criteria are as follows: the patients did not have other cancers except liver cancer.

### 2.2. MRI Examination

1.5 T superconducting MRI scanner and a 12-unit body array coil were adopted, and the scanning range was from the top of the diaphragm to the lower border of the liver. All selected patients completed T2-weighted imaging (T2WI) and T1-weighted imaging (T1WI) positive and negative phase and MRI-DWI and dynamic contrast-enhanced (DCE) sequence scans. Before the enhancement scan, the plain scan images were collected firstly; and the arterial phase, portal vein phase, and equilibrium phase images were collected 14 s after the enhancement. Images were collected to evaluate the number, size, and location of recurrent lesions in each phase of MRI enhancement.

### 2.3. Observation Indicators

The patients were followed up 3 months after the surgery to analyze the recurrence of liver cancer. The postoperative incision healing time, healing effect, and the need for secondary suture were analyzed and compared between the two groups. According to the *Diagnostic Standards for Nosocomial Infections of the Ministry of Health*, surgical wound healing standards could be determined as 3 grades [16]: grade I: good healing and no redness, swelling, induration, exudation, and pain; grade II: normal healing, with inflammation in the healing area, such as redness, induration, hematoma, and effusion, but no suppuration; and grade III: poor healing, incision was purulent, and incision drainage was required.

### 2.4. Retinex Algorithm

In 1963, E. Land firstly proposed the Retinex theory. After more than 40 years of development and improvement, the Retinex algorithm has become one of the most commonly used image enhancement methods. The principle was expressed as follows:

(1) $$\begin{array}{c} I\left(x,y\right)=S\left(x,y\right)∙R\left(x,y\right). \end{array}$$

In the above equation, (*x*, *y*) was the pixel index, and *I*(*x*, *y*) was the input image; *S*(*x*, *y*) referred to the ambient brightness, that is, the illumination component was the most direct factor affecting the dynamic range of the image; and *R*(*x*, *y*) represented the reflection component of the object. This decomposition can remove the illumination influence of the background light and the front light in the image. The principle of the Retinex algorithm was given as shown in Figure 1.

The core technology of image enhancement of this algorithm was to estimate the illuminance image *S*(*x*, *y*) from the original image *I*(*x*, *y*) and then calculate the reflection amount *R*(*x*, *y*) of the object according to the Retinex theory. In this study, the path-based Retinex algorithm was adopted, which referred to the most traditional algorithm and its improved algorithm. The path-based Retinex algorithm was mainly classified into three categories according to the different ways of selecting the path in the illumination estimation:

I. The theoretical basis of the random path Retinex algorithm was to randomly select a path between the start point *S* and the end point *E*. It was assumed that this path past through *n* pixels, and the pixel values of these points were {*p*_1_, *p*_2_, ⋯, *p*_*n*_}, using successively multiplied *n* pixels for brightness comparison to express the relative light-dark relationship:

(2) $$\begin{array}{c} \frac{E}{S}=T\left(\frac{p_{2}}{p_{1}}\right)\times T\left(\frac{p_{3}}{p_{2}}\right)\times \cdots \times T\left(\frac{p_{n}}{p_{n-1}}\right). \end{array}$$

In the above equation, *T*(*x*) was the threshold function, and its expression was given as follows:

(3) $$\begin{array}{c} T\left(x\right)=\left\{\begin{array}{cc} x, & \text{if }1-T\leq x\leq 1+T,\\ 1, & \text{if other}. \end{array}\right. \end{array}$$

With equation (3), the brightness relationship between the starting point and the ending point pixels can be calculated. The visual characteristics of the human eye can be simulated by a logarithmic function, so the logarithm of both sides of equation (3) can be obtained:

(4) $$\begin{array}{c} \log\left(\frac{E}{S}\right)=\log\left[T\left(\frac{p_{2}}{p_{1}}\right)\right]+\log\left[T\left(\frac{p_{3}}{p_{2}}\right)\right]+\cdots +\log\left[T\left(\frac{p_{n}}{p_{n-1}}\right)\right]. \end{array}$$

The value of log(*E*/*S*) was obtained by summing log[*T*(*p*_*i*_/*p*_*i*−1_)]. The function *T*(*x*) was converted to *T*′(*x*), and the expression was as follows:

(5) $$\begin{array}{c} \log\left(\frac{E}{S}\right)=\overset{n}{\underset{i=2}{\sum }}T^{\prime }\left(\log\frac{p_{i}}{p_{i-1}}\right)=\overset{n}{\underset{i=2}{\sum }}T^{\prime }\left(\log p_{i}-\log p_{i-1}\right). \end{array}$$

The algorithm selected the pixels on a one-dimensional random path to compare the brightness with the original pixels, the number of comparisons with the pixels in the original pixel area was small, and the illumination factor cannot be accurately estimated, so the enhanced image effect was not good. The algorithm was sensitive to the selected starting point and path. Different initial point and path selection would result in completely different enhancement results, and it was not easy to control the output results.

II. McCann's Retinex algorithm was an improvement based on the above algorithm. The algorithm selected a spiral path for comparison between pixels and used multiple iterations to reduce the influence of light factors on the original image. The number of pixels selected near the target pixel was relatively large, while the number of selected places at a distance was relatively small. This was determined by the smooth nature of the image, and points closer to the target pixel were more likely to have greater correlation. The algorithm firstly started the comparison from the farther pixels, the iterative comparison direction was rotated 90° clockwise, the distance was half of the previous time, and the target pixel stopped. Each iteration process was divided into the following four steps: proportion, product, reset, and average.

The input image *r*(*x*, *y*) was initialized as a brightness image, defined as *r*_0_(*x*, *y*), and the initial point was (*D*, 0). *D* referred to the conversion operator, whose size was determined by the length and width of the input image, and its expression was as follows:

(6) $$\begin{array}{c} D=2^{\left\lfloor \log_{2}\min\left(\text{rows},\text{cols}\right)-1\right\rfloor }. \end{array}$$

After a comparison, it was rotated 90° clockwise, the distance was halved, and the conversion operator was *D* = −*D*/2. At this time, the comparison was continued until |*D*| < 1. The iteration equation was as follows:

(7) $$\begin{array}{c} r_{n+1}\left(x,y\right)=\frac{r_{n}\left(x,y\right)+r_{n}^{\prime }\left(x,y\right)}{2}, \end{array}$$

(8) $$\begin{array}{c} r_{n}^{\prime }\left(x,y\right)=r_{n}\left(x,y\right)+∆l\;r_{n}\left(x,y\right)+∆l\leq \max, \end{array}$$

(9) $$\begin{array}{c} r_{n}^{\prime }\left(x,y\right)=\max\;r_{n}\left(x,y\right)+∆l\leq \max. \end{array}$$

In the above three equations, *r*_*n*_(*x*, *y*) was the result of the previous iteration, △*l* was the brightness difference between the compared pixels, max referred to the maximum value of the pixel in the input image, and *r*_*n*+1_(*x*, *y*) represented the final output result after *n* iterations. However, this algorithm was not efficient enough, so Funt et al. proposed the McCann99 algorithm based on the Gaussian pyramid model. The calculation process was roughly the same as the Frankle-McCann algorithm. The difference was that the algorithm used the pyramid model to compare the unit pixel and the 8 pixels in the 3 × 3 neighborhood with each pixel as the center from top to bottom and estimate the brightness value of each pixel, thereby inferring the reflection component. As the number of iterations increased, the input result calculated for each layer was interpolated to make the result of this layer the same size as the next layer and so on until the *n* + 1 calculation was completed.

For each layer operation of the pyramid, below equation was applicable:

(10) $$\begin{array}{c} r_{n}\left(x,y\right)=r_{n}\left(x,y\right)+s_{n}\left(x,y\right)-r_{n}\left(x+∆x,y+∆y\right)\;r_{n}\left(x,y\right)<\max, \end{array}$$

(11) $$\begin{array}{c} r_{n}\left(x,y\right)=\max r_{n}\left(x,y\right)\geq \max. \end{array}$$

In the above two equations, *s*_*n*_(*x*, *y*) was the input image pixel value of the *n*-th layer,  *r*_*n*_(*x*, *y*) referred to the output image pixel value of the *n*-th layer, and max represented the maximum value of *r*_*n*_(*x*, *y*). When the iteration result exceeded *r*_*n*_(*x*, *y*), it should be reset to max. ∆*x* and ∆*y* were the offsets in the neighborhood of the pixel (*x*, *y*).

III. Retinex algorithm based on center surround included the following algorithms.

The single-scale Retinex (SSR) algorithm could be expressed as follows:

(12) $$\begin{array}{c} \log R\left(x,y\right)=\log I\left(x,y\right)-\log\left(F\left(x,y\right)*I\left(x,y\right)\right). \end{array}$$

In equation (12), *I*(*x*, *y*) was the input image signal, *R*(*x*, *y*) referred to the output image, ∗ was the convolution symbol, and *F*(*x*, *y*) represented the center surround function. In the SSR algorithm, *F*(*x*, *y*) was the Gaussian filter function, which was expressed as follows:

(13) $$\begin{array}{c} F\left(x,y\right)=K∙e^{-\left(x^{2}+y^{2}\right)/\sigma^{2}}. \end{array}$$

In the equation above, *σ* represented the scale parameter of the Gaussian function, which was directly proportional to the sharpness. *K* was a normalization parameter, so the below equation could be obtained:

(14) $$\begin{array}{c} \int \int F\left(x,y\right)dxdy=1. \end{array}$$

It can be known from equation (12) that the SSR algorithm used the convolution principle to estimate the image illuminance change, subtracted the illuminance image from the original image to reduce the impact of illumination on the original image, and retained the reflected light imaging of the object, thereby meeting the need for image enhancement. For the single-scale Retinex algorithm, *σ* was the only parameter of the Gaussian filter (called the scale parameter). In order to ensure that the dynamic range was compressed while enhancing the contrast, it was very important to choose a suitable *σ*. In order to balance these two enhancement effects, the value range of *σ* is generally [80,120].

In order to make the output image reasonably mapped to the display range of the monitor, one of the solutions was adaptive contrast gain, which directly affected the quality of the output image. The mathematical equation was as follows:

(15) $$\begin{array}{c} R^{\prime }\left(x,y\right)=255\times \frac{R\left(x,y\right)-R_{\min}}{R_{\max}-R_{\min}}. \end{array}$$

In the above equation, *R*′(*x*, *y*) was the output image after linear grayscale stretching, *R*(*x*, *y*) referred to the enhanced image after SSR algorithm, and *R*_max_ and *R*_min_ were the maximum and minimum of the original image, respectively.

The basic principle of the multiscale Retinex (MSR) algorithm was the same as that of the SSR algorithm, which was a further optimization of the SSR algorithm theory. The MSR algorithm just introduced multiple scales on the basis of the SSR algorithm to calculate the SSR algorithm at the same time and then performed a weighted average of the calculation results. The output result expression was as follows:

(16) $$\begin{array}{c} R_{i}\left(x,y\right)=\overset{N}{\underset{n=1}{\sum }}W_{n}\left(\log I_{i}\left(x,y\right)-\log\left[F_{n}\left(x,y\right)*I_{i}\left(x,y\right)\right]\right). \end{array}$$

In the above equation, *i* represented the band number, and *i* = 1, 2, ⋯, *N*; *i* generally takes 1 or 3, representing grayscale images and color images, respectively. In color images, *R*_*i*_(*x*, *y*) represented the output image that has been enhanced in the three color spaces of R, G, and B; *I*_*i*_(*x*, *y*) represented the original image in the three color spaces of R, G, and B; *N* referred to the number of scales; *W*_*n*_ represented the weight of the *n*-th scale. Combining the enhancement results of three different scales in the multiscale Retinex algorithm can simultaneously obtain the advantages of the single-scale Retinex algorithm with high, medium, and low scales. The enhancement effect was ideal and the algorithm complexity was low. So when *k* = 3, *W*_1_ = *W*_2_ = *W*_3_ = 1/3 and *σ*_1_ < 50, 50 < *σ*_2_ < 100, *σ*_3_ > 100.

The MSR algorithm combined three different scale filtering effects on the basis of the SSR algorithm, which can not only maintain the color consistency of the image but also compress its dynamic range, so it was suitable for image sets that need to be enhanced in different application backgrounds. Although compared with the SSR algorithm, the enhancement effect of MSR on the color image had been significantly improved, but the color cast phenomenon still occurred.

Multiscale Retinex algorithm with color restoration (MSRCR algorithm) introduced a color restoration factor *C*, used the proportion of the input image in the three color channels to calculate the color restoration factor, and then adopted the color restoration factor to adjust the color of the output image to solve the bias color. The equation of the color restoration factor *C* was shown as follows:

(17) $$\begin{array}{c} C_{i}\left(x,y\right)=f\left(\frac{I_{i}\left(x,y\right)}{\sum_{i=1}^{3}I_{i}\left(x,y\right)}\right). \end{array}$$

In equation (17), *I*_*i*_(*x*, *y*) was the gray value of the original image *I* at the pixel point (*x*, *y*) in the *i*-th color channel, *f* was the mapping function, and *C*_*i*_(*x*, *y*) referred to the color restoration factor in the *i*-th color channel.

(18) $$\begin{array}{c} C_{i}\left(x,y\right)=\beta \times \log\left(a\times \frac{I_{i}\left(x,y\right)}{\sum_{i=1}^{3}I_{i}\left(x,y\right)}\right). \end{array}$$

After equation (18) was added to the MSR algorithm model, the algorithm model of MSRR can be obtained:

(19) $$\begin{array}{c} R_{i}\left(x,y\right)=\overset{N}{\underset{n=1}{\sum }}C_{i}\left(x,y\right)W_{n}\left(\log I_{i}\left(x,y\right)-\log\left[F_{n}\left(x,y\right)*I_{i}\left(x,y\right)\right]\right). \end{array}$$

In equation (19), *i* was the R, G, and B color channels, and *I*_*i*_(*x*, *y*) was the gray value of the original input image *I* at the *i*-th color channel pixel (*x*, *y*); *R*_*i*_(*x*, *y*) referred to the gray value of the reflection component *R* at the pixel point (*x*, *y*) in the *i*-th color channel, *N* represented the number of scales; *W*_*n*_ represented the weight assigned by the *n*-th scale, and the weight was generally set as the equal values; *C*_*i*_(*x*, *y*) was the color restoration factor of the *i*-th channel; ∗ referred to the convolution operation; and *F*_*i*_(*x*, *y*) was the Gaussian wrap function.

The MSRCR algorithm solved the serious color cast problem that occurred when the MSR algorithm enhanced color images. The introduction of color restoration factors effectively eliminated the color distortion of color images and coordinated the weight ratio between each color channel.

### 2.5. Image Enhancement Quality Evaluation

The quality of the enhanced image can be evaluated simultaneously through subjective and objective evaluation methods. In this study, two objective quality evaluation methods, namely, peak signal-to-noise ratio (PSNR) and structural similarity (SSIM), were selected, and the images enhanced by the five algorithms were compared. The expression was as follows:

(20) $$\begin{array}{c} \text{MSE}=\frac{1}{e\times Q}\overset{e}{\underset{i=1}{\sum }}\overset{Q}{\underset{j=1}{\sum }}{\left(M\left(i,j\right)-N\left(i,j\right)\right)}^{2}, \end{array}$$

(21) $$\begin{array}{c} \text{PSNR}=10\log_{10}\left(\frac{{\left(2^{n}-1\right)}^{2}}{\text{MSE}}\right). \end{array}$$

In the above two equations, MSE represented the mean square error of the current image *M* and the reference image *N*; and *e* and *Q* were the height and width of the image, respectively. The unit of PSNR was dB, and the larger the value, the more serious the image distortion.

SSIM is an image quality evaluation index that combines three aspects of contrast, brightness, and structure. It is often used in medical image evaluation. Its expression was as follows:

(22) $$\begin{array}{c} l\left(M,N\right)=\frac{2\mu_{M}\mu_{N}+C_{1}}{\mu_{M}^{2}+\mu_{N}^{2}+C_{1}}, \end{array}$$

(23) $$\begin{array}{c} l\left(M,N\right)=\frac{2\sigma_{M}\sigma_{N}+C_{2}}{\sigma_{M}^{2}+\sigma_{N}^{2}+C_{2}}, \end{array}$$

(24) $$\begin{array}{c} s\left(M,N\right)=\frac{\sigma_{MN+}C_{3}}{\mu_{M}\mu_{N}+C_{3}}. \end{array}$$

In equations (22)–(24), *μ*_*M*_ and *μ*_*N*_ represented the mean values of images *M* and *N*, respectively; *σ*_*M*_ and *σ*_*N*_ represented the variances of images *X* and *Y*, respectively; and *σ*_*MN*_ referred to the covariance of images *M* and *N*. *C*_1_, *C*_2_, and *C*_3_ were constants. In order to avoid the case where the denominator is zero, usually *C*_1_ = (*K*_1_ × *L*)^2^, *C*_2_ = (*K*_2_ × *L*)^2^, and *C*_3_ = *C*_2_/2. Generally, *K*_1_ = 0.01, *K*_2_ = 0.03, and *L* = 255. The SSIM expression was given as follows:

(25) $$\begin{array}{c} \text{SSIM}\left(M,N\right)=l\left(M,N\right)∙c\left(M,N\right)∙s\left(M,N\right). \end{array}$$

The value range of SSIM was in [0,1]. The larger the value, the smaller the image distortion.

### 2.6. Statistical Analysis

The SPSS22.0 software was adopted to perform data analysis to evaluate the efficacy of diagnostic methods. Measurement data between groups were represented by (*x* ± *s*), *t* test was performed, count data was represented by %, and *χ*^2^ test was performed. *P* < 0.05 indicated that the difference was statistically meaningful.

## 3. Research Results

### 3.1. Image Enhancement Quality Evaluation

Experiments were performed with brain MRI images, and comparative test results were given. Compared with traditional MRI, MRI based on Retinex algorithm showed clearer imaging, as shown in Figure 2. For the detection of three different image samples, the PSNR values of conventional MRI were 52.326, 60.942, and 54.677, respectively; and the SSIM values were 0.6217, 0.7539, and 0.5193, respectively. Based on the Retinex algorithm, the PSNR values were 62.168, 68.021, and 63.219, respectively; and the SSIM values were 0.7591, 0.8924, and 0.7196, respectively (as shown in Figures 3 and 4).

### 3.2. Detection Results of Different Methods for Postoperative Recurrence of Liver Cancer

A total of 48 cases with recurred liver cancer in 70 patients with liver cancer treated by laparoscopy in the postoperative reexamination, of which 31 were single lesions and 17 were multiple lesions. The lesions were 0.36-1.0 cm, with an average of 0.48 ± 0.14 cm. There were 18 cases with lesions in segment VIII, 11 cases with lesions in segment VI, 7 cases with lesions in segment VII, and 6 cases, 4 cases, and 2 cases in lesions in segments V, IV, and II, respectively. The detection results of different methods showed that the sensitivity, specificity, and accuracy of the detection of recurrent lesions in group A were 63.40%, 86.90%, and 78.60%, respectively. The sensitivity, specificity, and accuracy of detection of recurrent lesions in group B were 82.70%, 98.50%, and 93.20%, respectively. The difference between the two groups was statistically significant (*P* < 0.05). The specific results are shown in Figures 5 and 6.

### 3.3. Comparison of Wound Healing between the Two Groups of Patients

The average healing time of incisions in group D was significantly shorter than that in group C (*P* < 0.05). The results are shown in Figure 7.

The healing rates of grades I, II, and III in the study group were 88.57%, 8.57%, and 2.86%, respectively, while those in the control group were 45.71%, 40.00%, and 14.29%, respectively. The difference between the two groups was statistically significant (*P* < 0.05), as shown in Figure 8.

The second suture represented the suture of the granulation wound. Infected wounds and some purulent wounds that cannot be sutured or sutured were opened. The wound was sutured after normal granulation growth, clean wounds, and few bacteria in the secretions. The results showed that there were 2 cases of secondary suture in group D and 4 cases in group C. The test group was better than the control group in terms of probability, but *P* > 0.05 was found after statistical analysis. The result is shown in Figure 9.

## 4. Discussion

With the development of laparoscopic technology, most of the current hepatobiliary surgery can be replaced by laparoscopic surgery. Clinically, the commonly used follow-up methods after hepatobiliary surgery include ultrasound, CT, hepatic angiography, MRI, and radionuclide [17]. Among them, MRI shows high soft tissue resolution, multiparameter, multisequence imaging, and clear imaging. Studies have shown that the specificity and sensitivity of MRI examination are good, and it has good application value [18]. In addition, how to ensure good healing of the postoperative incision is one of the concerns of surgical operations. In the process of surgical wound healing, common complications such as fat liquefaction, subcutaneous effusion, and incision infection are prone to occur. These complications may delay wound healing and increase the pain and economic burden of patients [19]. Therefore, it is very important to promote wound healing and reduce wound healing delay caused by factors related to wound healing obstacles.

In this study, laparoscopic hepatobiliary surgery patients were selected as the research objects to explore the application value of MRI based on image enhancement algorithm in postoperative recovery and the influence of drainage tubes on surgical wound healing. The results showed that, taking brain MRI images as an example, MRI based on Retinex algorithm showed clearer imaging than traditional MRI. The PSNR values of conventional MRI were 52.326, 60.942, and 54.677, respectively; and the SSIM values were 0.6217, 0.7539, and 0.5193, respectively. Based on the Retinex algorithm, the PSNR values were 62.168, 68.021, and 63.219, respectively; and the SSIM values were 0.7591, 0.8924, and 0.7196, respectively. It can be concluded that the MRI imaging effect based on Retinex algorithm was better than conventional MRI. The detection results of different methods showed that the sensitivity, specificity, and accuracy of the detection of recurrent lesions in group A were 63.40%, 86.90%, and 78.60%, respectively. The sensitivity, specificity, and accuracy of the detection of recurrent lesions in group B were 82.70%, 98.50%, and 93.20%, respectively. The difference between the two groups was statistically significant (*P* < 0.05). This shows that MRI based on the image enhancement algorithm has a better effect on the detection of postoperative recovery of patients [20].

Compared with group C without subcutaneous drainage tubes, the average healing time of patients in group D was significantly shorter, and the healing rate of different grades of incisions was also significantly improved, showing statistically significant differences (*P* < 0.05). There are similar reports that placing drainage tubes under the skin facilitates the drainage of blood and fluid from the incision, thereby reducing excessive inflammation and promoting wound healing [21]. There were 2 cases of secondary suture in group D and 4 cases of second suture in group C. The test group was better than the control group in terms of probability. However, the statistical analysis showed *P* > 0.05; this may be related to the small number of subjects included in this study, so it has to be further studied. In short, poor wound healing may cause harm to the patient's body and mind and increase the patient's pain and financial burden. For hepatobiliary surgery patients with wound healing barriers, the preventive placement of subcutaneous drainage tubes is beneficial to improve the healing rate of the incision in grade A. This operation is simple, convenient, and low cost and does not increase patient suffering, so it is worthy of clinical application.

## 5. Conclusion

The MRI based on the Retinex algorithm was compared with the traditional MRI imaging results in the image enhancement algorithm. Studies have shown that MRI based on the image enhancement algorithm had a better imaging effect in postoperative recovery evaluation, and the detection rate of tissue abnormalities was higher. Comparison whether the patient had placed drainage tubes after surgery revealed that drainage tubes can effectively promote the healing of postoperative incisions and have clinical promotion value. However, the number of patients included in this study was small, and further research was needed for the accuracy of the results.

## Figures and Tables

**Figure 1:** Principle diagram of Retinex algorithm.

**Figure 2:** Comparison of MRI imaging with different methods. (a) Original image, (b) conventional MRI results, and (c) MRI results based on Retinex algorithm.

**Figure 3:** Comparison of PSNR values of different algorithms.

**Figure 4:** Comparison of SSIM values of different algorithms.

**Figure 5:** Comparison of the detection results of recurrent lesions by different methods. ^∗^Compared with group A, *P* < 0.05.

**Figure 6:** Evaluation of the detection results of recurrent lesions by different methods. ^∗^Compared with group A, *P* < 0.05.

**Figure 7:** The effect of drainage tubes on wound healing time. ^∗^Compared with group C, *P* < 0.05.

**Figure 8:** The effect of drainage tubes on wound healing. ^∗^Compared with group C, *P* < 0.05.

**Figure 9:** The effect of drainage tubes on the secondary suture of incision. ^∗^Compared with group C, *P* < 0.05.

## Data Availability

The data used to support the findings of this study are available from the corresponding author upon request.
